The article "Reading Game Sport from the Perspective of Sociology of Knowledge" was published in 2022. Journal: J Environ Public Health.

# Reading Game Sport from the Perspective of Sociology of Knowledge

**DOI:** 10.1155/2022/3711900

**Published:** 2022-07-04

**Authors:** Peng Shao, Han Yu, Zimu Xu

**Affiliations:** ^1^College of Humanities, Zhejiang University of Technology, Hangzhou, China; ^2^School of Journalism and Communication, Tsinghua University, Beijing, China

## Abstract

The evolution of media technology has not only changed readers' reading ways and reading habits but also tried to reshape their social behaviour. From the perspective of sociology of sustainable knowledge, this essay explores the impacts of technological change on reading through the framework of activity theory. It is found that digital reading is of increasing characteristics of “front stage” performance and reading anxiety in society, and sustainable knowledge anxiety began to spread. The research shows that the existing digital reading mode is actually the consumption of media, which is not conducive to the transmission and production of sustainable knowledge. Also, with the further development of technology, reading will open up a new chapter. The wisdom of human symbiosis will be infinitely stored and strive toward the era of global brain, which will help to better inherit sustainable knowledge and activate the vitality of sustainable knowledge production.

## 1. Introduction

In recent years, with the development of intelligent media, digital reading occupies most of the reading market. Every technological revolution is fraught with anxiety and fear, but it also ushered in opportunities and space for development. The latest figures show that, in 2019, China's adult national digital reading rate was 79.3 percent, which is 3.1 percentage points from the last year [1]. Reading media such as smartphones, tablets, and e-book readers are increasingly embedded in people's daily work and life, and readers' reading habits are increasingly influenced by the Internet and new media; “Reading on-screen” has become a unique “landscape” of modern society. The ecological relationship between reading media and readers, which influences and constructs each other, not only changes the carrier and form of reading materials but also changes the reading behaviour and thinking mode of readers derived from traditional paper reading.

Reading relies not only on oral language abilities but also on several executive functions. Considering their importance for literacy, training executive functions particularly, attentional control has been suggested as a promising way of improving reading skills [2]. An educational game tool in form of word tree was developed that did not only improve children's reading ability but also create happiness to learn [3]. Participation in the good behavior game improves children's rule compliance, general behavior, reading skills, and social inclusion [4]. Among them, we can highlight the use of gamification and game-based learning to motivate students towards learning to read and write [5]. Reading Turbo was integrated in a comprehensive phonics-based reading curriculum [6]. The aims of the study were to examine whether the game would advance children's word reading efficiency and to determine the extent to which prereading capacities and in-game mechanisms could explain individual variation in responsiveness to the game [7]. The gamification of mobile reading is driven by technology and increased nonutilitarian activities of human beings [8]. Mobile reading also generates fun through mechanism design and element matching to help users immerse themselves in it and achieve preset goals [6].

Although there exists extensive research on digital reading itself in the academic circles of our country, but the social impact caused by intelligent media has little attention. There is no consensus on how the media should be combined with reading in order to achieve better sustainable knowledge transmission and promote sustainable knowledge production. Therefore, there is a lack of empirical research on the current situation of national reading and the exact relationship between media technology and readers' social behaviour. How to make technology better realize sustainable knowledge production and cultural inheritance in the process of technology evolution has become a problem that needs attention of the whole society.

## 2. Related Works

As for the definition of sustainable knowledge, most scholars agree with Plato's view of sustainable knowledge in the Theaetetus that “sustainable knowledge is a true and verified belief” [9]. The history of western philosophy tradition tends to view epistemology as the theory of sustainable knowledge, so the classification of sustainable knowledge is regarded as an extremely complex cognitive activity, and different epistemists have different classification methods for sustainable knowledge.

The social sustainable knowledge school, comparing the stages of social development with those of sustainable knowledge development, holds that all sustainable knowledge, thought, intuition, and all forms of sustainable knowledge have sociological characteristics [10]. Meaningful experience is, first of all, mediated by social relations, which has an effect on the character of thought and sustainable knowledge [11]. From the point of view of sustainable knowledge creation, the creation of new sustainable knowledge is a complicated process, which can be accomplished only by establishing the connection and comprehension with the existing sustainable knowledge (i.e., “presustainable knowledge”) and realizing the internalization [12]. The main social process determines the spiritual life. When we study the role of thought, we should examine the social group behind the thought. Social economy and social life not only determine the generation of modern thought but also influence the form, structure, and content of spiritual products. The thoughts of the individual have much to do with the interest and purposes of his group [13].

Based on the theory of need, this essay adopts the research framework of the activity theory. From the perspective of the sociology of sustainable knowledge, the authors conducted an electronic questionnaire survey of 1,003 readers and three rounds of deep interviews with 22 readers with certain reading habits. This essay investigates the reading style, reading motivation, reading time and frequency, reading content, and reading situation of the audience and analyzes the reading behaviour of the audience with different age, income, educational background, and professional status. This essay analyzes the reading habits of the readers under the background of the change of the digital reading mode after learning about the choice of reading content, the characteristics of reading behaviour, the preference of reading media, and the changes of reading environment. Based on a large number of reading surveys and media research literature at home and abroad, this paper further explores the social impact of the digital reading mode, mainly including the readers' cognition, identity, and sustainable knowledge acquisition effect.

## 3. Research Methods

### 3.1. Questionnaire Method

Preparations for the survey were made from November 2018, and they lasted five years from the thirteenth to the seventeenth National Reading Survey results. We also collected and analyzed the reading survey questionnaires by the SPSS 21 statistic analysis tool. The questionnaire was distributed in many places in the country, including Shanghai, Xi'an, and Chongqing, to find out the possible reading problems in the society. Thus, it is determined that this time, using the mentality of the Reader Reading Situation Questionnaire Survey to carry on the question to set, Q1–Q10 are set up through the daily specific reading behavior of the reader (including reading time, reading content, and reading carrier) and reading purposes; Q11–Q14 are from the four dimensions of reading anxiety, namely, lack of reading time, information interference, lack of reading habits, and lack of systematic reading; Q15–Q17 are set up from the three dimensions of reading anxiety that reading cannot improve themselves, that is, they cannot remember what they read, cannot convert into their own thoughts, and cannot change their own behavior. The purpose of Q18–Q20 are to understand the impact of the two dimensions of sustainable knowledge anxiety (technological change and social competition) on readers; Q21–Q26 are part of the screening section and are used to obtain basic information about the subjects.

### 3.2. Interview Method

In order to accurately study more reading behavior and habit of readers with different background, 22 readers of different age, gender, education background, occupation, and rich reading experience were randomly selected. Indepth interviews were conducted on their daily reading behavior, reading scenes, and reading motivation. Each reader's interview is divided into three times, and 66 interviews are conducted for 22 readers. Each interview is limited to 1.5–2 hours, from the superficial to the deep and from the surface to the interior, trying to explain their reading behavior from the reader's own point of view. The orientation of the three interviews was as follows.

The first round of interviews is based on the individual reading experience of the interviewees. The purpose of the interviews is to understand the interviewees' cognition of the past reading behavior and to draw a general picture of the interviewees. The second round of interviews tracked participants' reading for a week, comparing them to self-reported reading behaviors. The third round is to listen to the interviewees' evaluation of their reading behaviors. One is listening to the readers' reaction on their previous reading behaviors, and the other is listening to the readers' statement about their future reading behaviors. The transcripts of the three interviews were archived in full, and the key contents were transcribed. Based on practical experience, the transcribed data of each interview ranged from 1,500 to 3,000 words, and each interviewee had no less than 5,000 words of interview data.

## 4. Research Findings

This research takes the activity theory as the concrete frame. The main factors in the activity theory are subject, object, and community, and the secondary factors are tools, rules, and division of labor. Among them, “subject” refers to the reader; “object” refers to the specific reading content; “community” refers to a whole formed in the process of reading; “rules” refers to the principles that readers must follow in reading, such as acquiring information and sustainable knowledge, realizing the transmission of sustainable knowledge and information, and “division of labor” refers to that, in socialized reading, members of the community are assigned their respective roles according to their roles.

### 4.1. Subject: Gender and Age Differences in Reading Behavior

The main body reading behavior analysis has mainly used the qualitative and quantitative methods. Through the analysis of questionnaires and interview texts, we find that male and female readers are similar in traditional reading, but the frequency and duration of male readers in digital reading are much higher than that of female readers (Table 1). At the level of reading duration, respondents prefer to read at night, and readers aged 20 to 29 spend the least time reading and are more likely to read on paper than any other age groups in (Table 2).

### 4.2. Object: News Information Is Still the Core of Reading

The analysis of reading object is mainly concerned with the preference of the reading subject to the reading content. The study found that most of the respondents preferred current affairs news (710 people) and entertainment information (404 people), which is closely related to the extensive entertainment in today's society. At the same time, life information is also the reading bias of the content (Figure 1). One of the reasons people choose to read is to obtain useful information of their lives.

*Q.* What kind of content do you like to read?

*A1.* Most of the time, I just binge-watch the news and watch some humorous content for fun. If there is a job evaluation or work needs to be promoted, I will also search for some professional books to read (M4).

It should be noted that when searching for reading contents, there are two kinds of reading subjects: active selection and passive selection. Active selection refers to readers' conscious search for the content, while passive selection refers to readers' reading based on the recommendation of big data.

Because the news content is more and short, and many times this is not the fundamental purpose of my reading, I will often browse. It is still necessary to keep up to date with news (M8).

### 4.3. Community: The Phenomenon of Reading for All Is Remarkable

The research of reading community mainly focuses on the comprehensive evaluation of readers' reading situation. Generally speaking, currently, the readers have better reading habits, but there are more obvious reading anxiety and sustainable knowledge anxiety. China is in a period of social transformation. With technological iteration and social competition, people are full of uncertainty and insecurity about their social status and prestige and are full of anxiety about their uncertain future and success [14]. On reading, 87.33% of the respondents agreed with “there are a lot of new technology, new sustainable knowledge that we have too much to learn” (Table 3); 48 percent agreed with the statement “I feel like everyone knows more than I do and I'm falling behind”; more than half agreed with the statement “I feel like my career is in trouble and I'm slow to improve myself.” Through cross analysis, we can find that the users who do not use digital reading at all have the lowest anxiety, and the people who are most prone to anxiety are those who read digital for less than 1 hour a day, followed by those who read digital for more than 3 hours a day. Users who read for 2-3 hours a day showed a relatively stable overall performance, but they also felt little anxiety.

### 4.4. Tools: Technology Integration Is Particularly Strong

The research on reading tools is actually the research on the media bias of reading subjects. With the development of mobile media, more and more reading media are available for readers to choose. The popularity and convenience of digital devices make more readers like digital reading. However, traditional reading relies on its authoritative, academic, and other irreplaceable qualities and still occupies a considerable proportion in readers' daily life. Text analysis of interview data shows that “digital,” “smart phone,” and “paper” are the most frequently discussed words (Figure 2).

When it came to media choices, 19 (86%) of the respondents said they were involved in both types of reading media and explained the reason why they choose it by comparing traditional reading with digital reading. This shows that the readers are choosing the reading carrier consciously according to the needs of their different reading scene. When we analyze the text, we find that the paper reading behavior, as a traditional reading, is often associated with “ritual sense” and “tactile sense.”

“Paper reading, for me, has a more pronounced sense of ritual, a sense of ritual that traditional reading allows me to touch paper, a sense of ritual that digital reading cannot replace. It was only through traditional reading that I understood more clearly that I was reading” (F6).

This psychology of the reader is a good reflection of the influence of the social environment on reading in an age when traditional reading is scarce. Paper reading makes the reader feel that he has enhanced his own charm. In terms of reading experience, traditional books allow the reader to concentrate on reading without the distraction of pop-up messages. This is the experience, painting on the book, that a digital reading cannot replace. From this, we can see that the traditional reading occupies an important position from the reading experience and reading effect in the majority of readers' mind. So why, in reality, are more and more people reading digitally?

“I enjoy traditional reading, but I definitely do more digital reading. Digital reading is easy to access, e-books are cheaper to download than paper books. The library is a bit far from home, and especially with the Kindle, I rely more on digital reading” (M4).

Paper reading usually requires a specific reading environment. Nowadays, with the explosion of social information, digital media has the timeliness and richness that traditional reading cannot reach. This naturally leads to a different division of labor between traditional and digital reading—digital reading for news, entertainment and traditional reading for professional sustainable knowledge. On the contrary, some readers show a preference for digital reading precisely because digital reading is not limited by time and space.

### 4.5. Division of Labor: Social Reading Is Becoming More Prominent

The research on the division of activities in reading is mainly concerned with the construction of reading and interpersonal relationship. In response to the question “How would you feel if you did not read for a long time?” 18 (82%) of the respondents said they would lose themselves and feel empty if they did not read for a long time; eight respondents (36 per cent) mentioned “social disconnection.” Obviously, for readers, the role of reading is not only in their own entertainment or self-improvement but also a part of social interaction.

“Without reading for a long time, I feel out of touch with society. If I cannot get information about social change from the Internet and mass media, I cannot keep up with the time and have nothing in common with the people around me. In this sense, reading also helps us to keep in touch with society. We get information from reading, which in turn helps us to build bridges with others. If a person does not read for a long time, he is easy to become behind the time, in the face of changing society, will have anxiety” (M1).

In addition to common social reading, reading exchanges between family members are also a notable phenomenon. In our indepth interview, there were 6 readers between 20 and 39 years old, who are female readers of primary childbearing age. Among them, 4 readers (67%) talked about children. The reading behavior of female readers in this age group tends to be significantly related to the upbringing of children.

“I'm raising a child for the first time, and every stage of a child's life is different. By reading books about parenting, I can learn more about it, learn from the experiences of others, and better deal with unexpected situations to take care of the baby” (F3).

## 5. Discussion

### 5.1. Media Revolution: Meeting the Diverse Reading Needs of Readers in the Context of Technological Evolution

Professor Wu Fei points out that technology is neither a means nor an end in itself when he studies the evolution of media technology. The original intention of creating media technology is for the freedom and liberation of “I” and “We,” so media is the essential condition of human's social existence [15]. Although digital reading has eroded some of the time of traditional reading, it also meets the needs of diversified reading and improves the comprehensive reading rate of the readers.

Chen Guangxing believes that we need to diversify our reading and reference frameworks in order to open up new possibilities. The real challenge is how to transform ourselves and how to diversify the fields and reference structures we identify with. Just as a healthy society needs multiple voices, so does a diverse reading medium. Different readers have different purposes for reading in different contexts, and a variety of reading styles help readers to acquire different types of sustainable knowledge and information.

From the reading media, reading can be divided into traditional reading and digital reading, and from the reading function, reading can be divided into social reading, shared reading, sustainable knowledge reading, and recreational reading. From the level of reading, reading can be divided into fragmented reading, systematic reading, and professional reading. Different media also have different bias, and the traditional reading scene is in a specific reading scene, with a desk and calm communication with the book, relying on personal experience to explain the orderly arrangement of text symbols. The content of its dissemination is often personalized, abstract, systematic, and serious, which meets the needs of readers' sustainable knowledge production, consumption, and promotion of their own competitiveness; digital reading transfers the private book page to the shared screen, as it is not limited by time and space and the content is usually popular, figurative, fragmented, and entertaining, meeting the needs of social and recreational readers [16]. Traditional reading, digital reading, or other reading are born with the needs of the reader and depend on the characteristics of the media to influence the reader's reading habits, building a diverse reading society.

Therefore, how to acquire sustainable knowledge is no longer a shackle that prevents readers from reading. How to weigh the importance of various types of sustainable knowledge in different situations and identify the sustainable knowledge that has the most value to guide them to support themselves to make timely decisions has become one of the most serious challenges in reading [17].

### 5.2. Digital Reading: A Seemingly Convenient Way of Acquiring Sustainable Knowledge in a Technological Package

The medium is an extension of man. With the transformation of social life by the development of communication technology, readers have an unprecedented illusion of “Liberation”: now, if you want to read a book, you do not need to go to the bookstore, just take out the Kindle and then you can download what you want; you do not even have to read line by line to get a general idea because you can know what is important on a page from someone else's notes, or you do not even have to read it by yourself and you can pay for the sustainable knowledge to see the best parts of a book that someone else has distilled. It is one thing to hear and read something, that is to say, we can simply know something, but it is another matter to think about what we have seen. Under the technology packing, taking the payment for sustainable knowledge as an example, many new sustainable knowledge dissemination methods seem to help the reader to obtain the sustainable knowledge more conveniently, but it actually has the latent interest demand of some groups, which has reflected these groups' values. In traditional reading, social factors influence readers' understanding of sustainable knowledge, while in digital reading, some interest groups are constructing readers' cognition and values, which is very harmful to cultural inheritance.

Sustainable knowledge has never been static, but it is a constantly changing process with the development of society and the evolution of ideas. Jiddu Krishnamurti once said that even though can become a shackle to the freedom of mind because all that is thought and thought is old. The value of reading lies in inscribing the crystallization of human thought civilization in the symbol, which has the character of defying the erosion of space and time, making it inherit and develop continuously and promoting the progress of society. In the process of sustainable knowledge transmission, sustainable knowledge and perception cannot be separated; otherwise, there will be false sustainable knowledge or perception [18]. In essence, digital reading is the consumption of media and the payment of services. It weakens the importance of sustainable knowledge itself consciously or unconsciously. Obviously, in the social evolution, the digital reading pattern presents the characteristic that we do not even need to consider, which is not beneficial for the independent thinking and new thoughts. The reading sustainable knowledge under this mode is constructed by the society, while the traditional reading emphasizes logic and order, opposes contradictory expression, and advocates calm, objective, rational, and abstract reading thinking. Only in this way can the reading form a balanced antagonistic force with the society and mutual construction of society. It can be said that traditional reading can more reflect the value of reading, create new sustainable knowledge, and achieve the transmission of sustainable knowledge, while digital reading is more inclined to different media on the record of sustainable knowledge.

### 5.3. Traditional Reading: A Truly Effective Way to Acquire Sustainable Knowledge in the Development of Society

The “sustainable knowledge” imagined by Plato is like the “seed” that the mind is born with. It is awakened through education or other means and germinates into sustainable knowledge [19]. The traditional sustainable knowledge production has brought up numerous human wisdom with scientific theory and philosophy thought, which profoundly transformed the world [20]. Along with the development of society, digital reading has also joined the agenda, but the effect is quite different.

In the digital age of reading, recommended reading, sharing, highlighting, and underlining all add to the fun of reading, but it is actually an output of ideas behind each recommendation. Reading platforms make commercial profits from quantity of flow. When the audience is gripped by technology, instead of relying on digital media for more autonomy, they fall into the trap of power. The possibility of a “gatekeeper” platform recommending a work to a majority of readers actually weakens the reader's right to choose. Under the control of media, most digital users read similar content, but the cognitive level of readers is different. The mismatch between the acquired sustainable knowledge and their own needs will not alleviate the anxiety of the readers, but will increase it; meanwhile, under the situations of group decision-making, the opinions or decisions of individuals often result in group consistency because of the influence of discussions among groups. In the long run, the readers sustainable knowledge structure and mode of thinking may be potentially regulated, and sustainable knowledge production is maintained at a similar level, which is not conducive to the creation and transmission of sustainable knowledge.

## 6. Conclusions

Polanyi calls ideal sustainable knowledge as “personal sustainable knowledge,” and accordingly, ideal sustainable knowledge production is a purely individual activity [21]. According to our original ideas, sustainable knowledge production is the activity and process that people pursue to realize their personal interest. Sustainable knowledge as the product of sustainable knowledge production can be objective only when it is a purely personal activity; on the other hand, if objective factors are involved in the process of sustainable knowledge production, sustainable knowledge itself may be adulterated with subjectivity and may lose its credibility. From paper reading to digital reading, from reading time to screen reading time, each kind of reading development process is an innovation-driven product and represents the development direction of reading. The role of technology will not be limited to connecting people and things with nonthings because technology comes from society and becomes a deep-rooted part of society. It will continue to work with mankind to build a better society and realize the redemption of the spirit of the times.

## Figures and Tables

**Figure 1:** Respondents' preference for reading content.

**Figure 2:** The word cloud chart of high-frequency words in interview data.

**Table 1:** Gender differences in reading behavior among different age groups.

	Male	Female
Tradition reading	27 times/875 min	16 times/865 min
Digital reading	47 times/932 min	10 times/600 min^1^
Tradition reading	15 times/680 min	28 times/1325 min
Digital reading	44 times/1835 min	36 times/1350 min^2^
Tradition reading	29 times/1501 min	33 times/905 min
Digital reading	49 times/2225 min	68 times/2255 min^3^
Tradition reading	18 times/520 min	18 times/685 min
Digital reading	75 times/3470 min	27 times/770 min^4^

^1^Gender differences in the use of reading media by readers aged 20–29. ^2^Gender differences in the use of reading media by readers aged 30–39. ^3^Gender differences in the use of reading media by readers aged 40–49. ^4^Gender differences in the use of reading media by readers aged 50–60.

**Table 2:** The temporal differences of reading behavior among different age groups.

Age	20–29		30–39		40–49		50–59	
Reading Media	Tradition	Digital	Tradition	Digital	Tradition	Digital	Tradition	Digital
Morning 6 : 00–12 : 00 (min)	365	292	620	730	590	940	575	855
Noon 12 : 00–18 : 00 (min)	240	200	670	820	730	990	240	1073
Evening 18 : 00–6:00 (min)	1135	1040	715	1635	715	1635	385	1635

**Table 3:** Cross table of digital reading time and sustainable knowledge anxiety factors.

*How much time do you speed reading digital books every day?*	*There are a lot of new technology, new sustainable knowledge that I have to learn*					Total
	*Totally agree*	*Agree*	*May be*	*Disagree*	*Totally disagree*	

Within an hour	62	141	20	14	5	242
An hour or two	124	100	38	1	1	264
Two or three hours	56	116	11	3	4	190
More than three hours	119	114	8	1	0	242
Barely read	19	25	14	6	1	65
Total	380	496	91	25	11	1003

*How much time do you speed reading digital books every day?*	*I feel like everyone knows more than I do and I'm falling behind.*					*Total*
	*Totally agree*	*Agree*	*May be*	*Disagree*	*Totally disagree*	
Within an hour	46	99	66	24	7	242
An hour or two	48	85	102	25	4	264
Two or three hours	22	44	90	14	20	190
More than three hours	28	75	110	27	2	242
Barely read	21	17	22	2	3	65
Total	165	320	390	92	36	1003

*How much time do you speed reading digital books every day?*	*I feel like my career is in trouble and I'm slow to improve myself.*					*Total*
	*Totally agree*	*Agree*	*May be*	*Disagree*	*Totally disagree*	
Within an hour	43	124	52	21	2	242
An hour or two	47	90	88	37	2	264
Two or three hours	20	78	64	28	0	190
More than three hours	35	70	62	71	4	242
Barely read	17	34	13	0	1	65
Total	162	396	279	157	9	1003

## Data Availability

The data used to support the findings of this study are available from the corresponding author upon request.
